This article has been retracted.

# Multimodal Medical Image Fusion of Positron Emission Tomography and Magnetic Resonance Imaging Using Generative Adversarial Networks

**DOI:** 10.1155/2022/6878783

**Published:** 2022-04-14

**Authors:** R. Nandhini Abirami, P. M. Durai Raj Vincent, Kathiravan Srinivasan, K. Suresh Manic, Chuan-Yu Chang

**Affiliations:** ^1^School of Information Technology and Engineering, Vellore Institute of Technology, Vellore 632014, India; ^2^School of Computer Science and Engineering, Vellore Institute of Technology, Vellore, 632 014 Tamil Nadu, India; ^3^Department of Electrical and Communication Engineering, National University of Science and Technology, Muscat, Oman; ^4^Department of Computer Science and Information Engineering, National Yunlin University of Science and Technology, Yunlin 64002, Taiwan; ^5^Service Systems Technology Center, Industrial Technology Research Institute, Hsinchu, Taiwan

## Abstract

Multimodal medical image fusion is a current technique applied in the applications related to medical field to combine images from the same modality or different modalities to improve the visual content of the image to perform further operations like image segmentation. Biomedical research and medical image analysis highly demand medical image fusion to perform higher level of medical analysis. Multimodal medical fusion assists medical practitioners to visualize the internal organs and tissues. Multimodal medical fusion of brain image helps to medical practitioners to simultaneously visualize hard portion like skull and soft portion like tissue. Brain tumor segmentation can be accurately performed by utilizing the image obtained after multimodal medical image fusion. The area of the tumor can be accurately located with the information obtained from both Positron Emission Tomography and Magnetic Resonance Image in a single fused image. This approach increases the accuracy in diagnosing the tumor and reduces the time consumed in diagnosing and locating the tumor. The functional information of the brain is available in the Positron Emission Tomography while the anatomy of the brain tissue is available in the Magnetic Resonance Image. Thus, the spatial characteristics and functional information can be obtained from a single image using a robust multimodal medical image fusion model. The proposed approach uses a generative adversarial network to fuse Positron Emission Tomography and Magnetic Resonance Image into a single image. The results obtained from the proposed approach can be used for further medical analysis to locate the tumor and plan for further surgical procedures. The performance of the GAN based model is evaluated using two metrics, namely, structural similarity index and mutual information. The proposed approach achieved a structural similarity index of 0.8551 and a mutual information of 2.8059.

## 1. Introduction

The process of image fusion combines the unique features and spatial attributes to generate single fused image using images from single or multiple modalities [1]. This is performed to improve the results of medical image analysis. The ultimate aim of multimodal medical image fusion is to retain the spatial feature of the image and to make the medical image analysis and disease diagnosis accurate and less time consuming [2]. Medical image fusion is found to be successful in multivarious fields, namely, image enhancement, medical image analysis, and surveillance. Medical image fusion helps in diagnosing and classifying disease with high accuracy [3]. The classical approach of medical image fusion is to perform medical image registration, which aligns the images obtained from multiple sources resulting in single enhanced output image obtained from two or more input images [4]. The ultimate goal in combining the multimodal images is to transform the images into highly informative and classifiable image. Some of its applications are classification of disease, weather prediction, and other operations related to military. Deep learning is found to be successful in many applications [5] like image fusion, segmentation [6], facial expression recognition [7], and other medical-related application [8]. Abbreviations presents the full forms used in this work.

With the advancement in technology highly reliable medical imaging tools and techniques like Magnetic Resonance Image, Positron Emission Tomography, and Computed Tomography, they have come up making the diagnoses of diseases accurate and less time consuming [9]. Positron Emission Tomography is not involved in the introduction of any medical instruments into the human body. Rather, it utilizes Positron Emitting Radioisotopes to generate multiple images based in tissue concentrations [10]. However, considering PET image alone has several drawbacks. The spatial resolution of PET images is very low making the medical diagnoses difficult. However, pathological and molecular information can be obtained from PET. Similarly, MRI provides regional change details in physiology, tissue composition, and hemodynamics functional information. Hence, performing the fusion of images from different or same modalities has become inevitable to obtain accurate results [11].  Figure 1 shows some of the medical diagnostic images used in recent times. Combining these images makes the resulting image information rich with features integrated from multiple modalities. Image fusion adds advantage of using combining all the important information from different images into one single fused image making the process of image analysis easier, quicker, and accurate. Also, image fusion technique enhances the spatial clarity of the fused image. The space occupied for storing individual images is greatly reduced when multiple images are fused together into single image.

MRI and CT images are structural images with higher resolution and anatomical structure [12]. PET and SPECT are functional images with lower resolution and functional information [13]. Several research works have already been proposed related to multimodal medical image fusion to overcome the drawbacks of single images from various modalities [14]. However, the existing approaches have their own advantages and disadvantages. Wavelet transform was one of the frequently used approaches for performing medical image fusion [15]. Few other approaches used to perform medical image fusion are discrete wavelet transform [16], stationary wavelet transform [17], redundancy wavelet transform, average method, principal component analysis, brovey method, and curvelet transform. However, technically, combining PET images with MRI images is challenging because of the existing incompatibility between magnetic field and the PET detectors. Also, some of the existing image fusion approaches presume that distortions follow Gaussian distribution leading to model mismatch problem. These issues are handled by using generative adversarial networks for combing PET and MRI images. Yet another challenge in combining PET and MRI images is that MRI image is a grey scale image while the PET image is a pseudocolored image.  Figure 2 shows various existing approaches adopted to perform image fusion. These approaches have several advantages and disadvantages. The main disadvantages of the existing approaches are the actual chromaticity of the diagnostic images which are not preserved. In order to overcome these drawbacks, medical image fusion is proposed using generative adversarial networks. Combining medical images has been proven successful for scientific and medical purposes especially oncology, cardiology, and neurology.

Combining PET and MRI images into a single image allows simultaneous acquisitions, though instinctively simple; it is technically more challenging than it appears to be [18]. It has been impossible to combine these two diagnostic images for several years because of their incompatibility between photomultiplier tube of PET and powerful magnetic field of MRI [4]. As a solution to this issue, it has been proposed to perform sequential PET-MRI scans for the patient and subsequent merging of this bimodality system for accurately fusing these diagnostic images. However, the process was complex and time-consuming. In order to overcome these issues and make the process simpler and less time-consuming deep learning-based approaches have been proposed to perform multimodal image fusion for medical diagnostics.

Brain tumor is collection of anomalous cells in a human brain affecting more than 15 million people every year [19]. It is considered a global health problem; timely prediction is necessary to prevent a medical condition to save lives [20]. Hence, detecting brain tumor at an early phase is necessary to provide timely medical intervention and prevent further complications [21]. The outcome can be improved by taking appropriate action on the warning signs of brain tumor. In recent times, brain images in modalities like computed tomography, MRI, and PET are used to evaluate the intensity of the stroke [22]. Deep learning models have proven successful in many medical applications. Hence, a deep learning-based robust model is proposed to utilize multimodal medical images to detect a brain tumor. Here, the proposed model performs multimodal medical image fusion to detect a brain tumor. Fusion of PET and MRI images are performed using generative adversarial networks to detect a brain tumor.

Behavioral disorder involves disorderly behavior in childhood or adolescence. Some of the frequently seen behavioral disorder in children are bipolar disorder, anxiety disorder, depression, bipolar disorder, learning disorder, conduct disorder, attention deficit hyperactivity disorder, oppositional defiant disorder, and autism spectrum disorder. Some of the childhood issues are related with family history and gender. The children with behavioral disorder express inability to obey rules, arguing recurrently, seeking revenge, and deliberately annoying others. The child may also express difficulty in concentrating, difficulty making friends, low self-esteem, and persistent negativity. The children with behavioral disorder may be given family therapy by a child psychiatrist.

The main contribution of the proposed work is that it models an effective image fusion technique using generative adversarial networks. The proposed approach adopts a novel dual discriminator approach to perform multimodal medical image fusion. The results display that the proposed approach is superior to the existing medical image fusion approaches in preserving the anatomical and functional information of the input images.

In this paper, the proposed model performs multimodal medical image fusion for combining multimodal brain images, namely, PET and MRI using generative adversarial network. The working flow of the paper in the following fashion.  Section 2 describes other works that are related to medical image fusion.  Section 3 describes the materials and methods adopted to perform medical image fusion, network architecture, and the loss function used in the proposed work.  Section 4 discusses about the experiments and the result.  Section 5 concludes the proposed work.

## 2. Literature Review

Multimodal medical image fusion acts as a potential tool for performing medical diagnosis and provide timely treatment for the diagnosed disease [23]. PET and MRI images are considered to be one of the most advanced imaging techniques in the medical field. A detailed and accurate assessment of a human subject can be made bringing together the molecular data presented by PET and the functional and morphological data presented by MRI. The fused image is capable of simultaneously providing high-resolution molecular, anatomic, and functional data allowing brain tumor analysis and segmentation in a single image examination. This fusion technique has also brought a massive progress in diagnosing cancer, its stages, and the response to the treatment [23]. Multimodal image fusion has made the detection of metastases easier, which was complex with individual image modalities.

Haddadpour et al. proposed an approach to combine PET and MRI images. The authors used a 2-dimensional HT and IHS to perform multimodal image fusion. The performance of the model is tested using performance metrics. Discrepancy evaluates the performance of the model in retaining the spectral features in the fused image. A higher spectral resolution is achieved with lower value of discrepancy. The discrepancy obtained using this method is minimum resulting in retaining spectral features. Also, the method achieved good average gradient resulting in retaining spatial features. The difference between overall performance and discrepancy represents the overall performance. Lower value of overall performance indicates a better fusion quality. The combination of 2-dimensional HT and HIS resulted in low overall performance [24].

Shahdoosti and Mehrabi proposed PET-MRI image fusion using dual ripplet II transform. Ripplet II transform suffers from shift variance problem. In order to overcome this issue, the authors proposed dual repplet II transform. The color and spatial information of the image is preserved using a weighing matrix. Dual ripplet transform is advantageous over ripplet II transform as traditional wavelet is used in ripplet II transform and complex wavelet is used in dual ripplet II transform. Also, dual ripplet II transform uses generalized radon transform. The proposed approach decomposes the input image into low-pass bands and then to high-pass bands. The proposed method used MRI images of good resolution and PET images that are colored images. The size of PET images was not the same as that of MRI images. MRI images were of size 256 × 256 while PET images where of size 128 × 128. So to match the size of PET and MRI images to perform fusion of images, PET images were upscaled to 256 × 256 pixels. The images were obtained from Harvard University website. The experiment used images of different disease categories, namely, coronal and Alzheimer's disease. The parameter settings were 0.03 for *λ*, 0.005 for *β*, and 0.001 for *ε*. The proposed approach preserved the functional features of PET image and anatomical details of MRI image. The model is evaluated using normalized weighted performance metric. The proposed model achieved 0.8771 normalized weighted performance metric [25].

Ouerghi et al. performed a fusion of PET-MRI images based on shearlet transform and a NN model. The proposed approach converted the input PET image into independent components. Both MRI and the transformed independent components of PET images are broken up into two bands, namely, the low frequency and high frequency. The nonsubsampled shearlet transform combines the low-frequency components. A simplified pulse coupled neural network model combined high-frequency components. The proposed model initially performed MRI and PET image registrations. The registered images are further normalized and then transformed into independent components. This is performed to separate the chromatic information and the illuminance of the input. The model is compared with other models using fusion quality index [26]. Du et al. performed the fusion of PET-MRI images using intrinsic image decomposition approach to decompose the images into 2 different components. It used two algorithms; one algorithm extracted the anatomical information of the image while keeping the noise level from the input low. Another approach performed summing up of the color details obtained from input image. The signal-to-noise ratio obtained from the proposed approach is very less in comparison with other models. The implementation of the model is compared with Bonferroni-Dunn and Friedmann tests. Though the proposed work performed reasonably good in combining the PET and MRI images, the proposed approach expressed dependencies of intrinsic image decomposition [27].

Liu et al. proposed a model to fuse medical image using multiresolution and nonparametric density models. The space registered input images are first generalized and then broke into different frequency components using contourlet transform. The model is evaluated using average cross entropy that calculates the difference between the input and the output. Lower value of average cross entropy results in better fusion. The clarity and spatial resolution of the resultant image is assessed using average gradient. When the value of average gradient high, it implies better spatial clarity. The proposed approach is compared quantitatively and qualitatively with six fusion methods on three classes of images, namely, Alzheimer's, normal, and neoplastic images of brain. The quality of the final fused image is assessed using five different metrics, namely, mutual information, edge intensity, average gradient, average cross entropy, and entropy. The proposed approach achieved 0.1558 cross entropy, 90.5 edge intensity, 9.166 average gradient, and 3.9 mutual information [28]. Tang et al. [29] obtained the neighborhood information to realize the focused and defocused pixels of the input image. Prabhakar et al. proposed medical image fusion using unsupervised deep learning model. Multimodal image fusion is performed using a generative adversarial network [30–32].  Table 1 shows the existing approaches in performing multimodal medical image fusion.

## 3. Materials and Methods

PET images are of low spatial resolution depicting the brain function. MRI images depicts the anatomy of brain and does not possess any functional details of the brain. Obtaining the necessary clinical information from a single image is practically not possible. Hence, to get accurate results of diagnosis, the diagnostic image should depict both spatial characteristics and functional information with no distortions. Hence, combining PET and MRI images would be a highly reliable diagnostic tool to perform image analysis. The image fusion should be performed in a way that the fused image retains the anatomic, functional, and structural details of the input images.

The primary goal of the proposed work is to combine the MRI image and PET image. The goal of generator in GAN is to generate the data distribution same as that of the input data. The goal of discriminator is to differentiate the output image from the original image. When the discriminator is not capable of differentiating the output image from the actual image, the generator has learnt the data. The goal of the GAN proposed in this model is to selectively retain the information present in the input images, namely, MRI and PET. The details retained are controlled by the hyperparameters.  Algorithm 1 represents the workflow of the proposed model in generating the fused image.

Given the input images PET and MRI, the whole process of image fusion is represented in Figure 3. To retain the functional details of PET and anatomical details of MRI, we formulated a novel model using GAN to fuse the given input images. The input images are concatenated and sent to the network generator. The output generated from the generator is a fused image *I*_fu_. The generated image *I*_fu_ represents the structural information of MRI *I*_mri_ and functional details of PET *I*_pet_. Followed by this, the output image *I*_fu_ and the input image is compared. The proposed approach establishes a min max game between generator and discriminator, and with more number of iterations the *I*_fu_ will contain more and more details from the input image. During the process of training, if the discriminator fails to distinguish between the actual and the generated samples, the generator is trained well. The generated image is then passed as input to the dual discriminator. One discriminator receives MRI image and combined image as the input and the other discriminator receives PET image and the fused image as the input. The discriminator *D*_*m*_ is trained to differentiate the generated image from the MRI image, while the discriminator *D*_*P*_ is trained to differentiate the output image from the PET image. The generator training with two discriminators is formulated as

(1) $$\begin{array}{c} \min\;G\;\max\;D_{M}D_{P}\;\left(G,D\right)=E\left[\log\;D_{M}\left(I_{\text{mri}}\right)\right]+E\left[\log\left(1-D_{M}\left(G\left(I_{\text{mri}},I_{\text{pet}}\right)\right)\right)\right]+E\left[\log\;D_{P}\left(I_{\text{pet}}\right)\right]+E\left[\log\left(1-D_{P}\left(G\left(I_{\text{mri}},I_{\text{pet}}\right)\right)\right)\right]. \end{array}$$

According to equation (1), the generator is trained to minimize the above equation and discriminator is trained to maximize the above equation.

The loss function of the proposed model is composed of two losses. One loss is from the generator, and the other loss is from the discriminator. The generator loss *L*_*G*_ represented by equation (1) is again composed of two components. The first component is the adversarial loss, which is the loss between the generator and the discriminator.

(2) $$\begin{array}{c} L_{G}=L_{\text{Adv}}+{\gamma L}_{\text{Inf}}. \end{array}$$

The second component in the generator loss *L*_*G*_ represents the information loss. Since the MRI image *I*_*g*_ has information related to anatomical details of brain and PET image, *I*_*q*_ has information related to function; it is enforced that the fused image *I*_*f*_ to represent similar functional and anatomical information as *I*_*q*_ and *I*_*g*_. *γ* is the parameter controlling the tradeoff between adversarial loss and information loss.

The architecture of generator in GAN is represented in Figure 4. The generator has five layer CNN with 3 × 3 filters in each of the layers. The value of stride in each of these five convolutional layers is set to one. The input to the generator is a PET-MRI concatenated image. The convolutional layers extract feature maps of input image. Batch normalization is used in generator architecture to make the model more stable. Leaky Relu is used in all the layers of the generator before the last layer, and tanh activation function is used in the last layer. Leaky Relu and Tanh are represented as follows:

(3) $$\begin{array}{c} \text{Leaky Relu}=\max\left(0.1x,x\right), \end{array}$$

(4) $$\begin{array}{c} \text{tanH}=\tanh\left(x\right). \end{array}$$

The architecture of the discriminator of GAN is represented in Figure 5. The discriminator has five layer CNN with 3 × 3 filters in the first four layers and 1 × 1 filter in the last layer. The value of stride in each of these five convolution layers is set to two. The discriminator is basically a classifier which first performs feature extraction and then performs classification. Batch normalization is used in the layers between the first and the last layers. Leaky Relu is used as the activation function in all the layers before the last layer, and tanh is used in the last layer. The last layer performs the classification which classifies the image as real or generated image. The flowchart of the proposed approach is represented in Figure 6.

## 4. Experiments and Results

The data for the proposed approach is obtained from the medical library of Harvard University, (http://www.med.harvard.edu/AANLIB/home.html). Pairs of MRI and PET data were obtained from the database. The database had MRI images of high resolution with size 256 × 256 and the PET images with size 128 × 128. In order to perform the fusion of images, PET images were resized to 256 × 256. Some of the sample PET images obtained from the database are represented in Figure 7, and sample MRI images obtained from the database are shown in Figure 8.

The result obtained from the proposed approach is represented in Figure 8.  Figure 9(a) shows the input MRI image, Figure 9(b) shows the input PET image, and Figure 9(c) shows the generated fused image. From the results obtained, it is clearly visible that the anatomical structure of MRI and functional details of PET are preserved in the resulting fused image.  Figure 10 shows the comparison of results obtained from the proposed approach and weighted averaging technique [36].

Table 2 shows the performance of the proposed approach in comparison with other existing approaches in performing medical image fusion. The performance of the proposed model is estimated using average structural similarity and mutual information. Average structural similarity is a metric that determines the similarity between two images and estimates the quality degradation after performing the image fusion. Mutual information is the metric that assesses the quantity of information that is being transferred from the input images and the source image.

(5) $$\begin{array}{c} \text{Mutual information},I\left(X;Y\right)=\Sigma_{x\epsilon X}\;\Sigma_{y\epsilon Y}p\left(x,y\right)\log\frac{p\left(x,y\right)}{p\left(x\right)p\left(y\right)}, \end{array}$$

where *p*(*x*) and *p*(*y*) are the marginal probability distribution functions of both the margins and *p*(*x*, *y*) is the marginal probability distribution.

(6) $$\begin{array}{c} \text{Structural similarity index},=\frac{1}{M}\overset{M}{\underset{J=1}{\sum }}Q\left(\left\{\left.i_{k}\left(j\right)\right)\right\},F\right), \end{array}$$

where *Q* is the correlation coefficient between the ground truth image and the fused image.

## 5. Conclusion

In the past few years, image fusion has been immensely used for several image-processing applications in various fields, particularly medical applications like retinopathy and brain tumor segmentation. The work presented a novel approach in performing medical image fusion using generative adversarial networks. The proposed approach efficiently captured the functional information from PET images and anatomical structure from MRI images and transformed them to the resulting fused image. The proposed approach generates fused images with less distortion and better structural information when compared to the existing approaches. The advantages of the proposed approach over the other existing approaches are that it can retain the textural information from the MRI image and the metabolic information from the PET image without losing pixel intensity. The performance of the proposed approach is evaluated using two metrics, namely, structural similarity index and mutual information. The proposed approach achieved a structural similarity index of 0.8551 and a mutual information of 2.8059. The results display that the proposed approach is superior to the existing medical image fusion approaches in preserving the anatomical and functional information of the input images. The work can be extended in performing the fusion of multimodal images with color. Also, the future work can incorporate other deep learning techniques and evaluate the performance using various other metrics. The work still needs to be improved to handle images with more noise.

## Figures and Tables

**Figure 1:** Medical image modalities.

**Figure 2:** Methods adopted to perform image fusion.

**Figure 3:** Architecture of the proposed approach for image fusion.

**Figure 4:** Generator architecture.

**Figure 5:** Discriminator architecture.

**Figure 6:** Flowchart of the proposed approach.

**Figure 7:** Sample PET images from the dataset.

**Figure 8:** Sample MRI images from the dataset.

**Figure 9:** Result obtained from the proposed approach.

**Figure 10:** Comparison of obtained fusion results with existing approach.

**Algorithm 1:** 

**Table 1:** Medical image fusion—existing approaches.

Modality	Work	Organ	Fusion technique	Approach
PET and MRI	[24]	Brain	2D Intensity Hue Saturation and Hilbert transform	PET and MRI image fusion using 2D Hilbert transform and Intensity Hue Saturation Fourier Transform is calculated for each of the input signals.
PET and MRI	[25]	Brain	Dual ripplet II transform	The proposed approach uses dual ripplet II transform as it uses complex wavelet transform. The color and spatial information of the images are preserved using weight matrix.
PET and MRI	[27]	Brain	Intrinsic image decomposition	Model based on intrinsic image decomposition are proposed to extract structural information from MRI and for obtaining color details from PET.
PET and MRI	[26]	Brain	Non-subsamples shearlet transform	The input images are registered and normalized and then transformed into independent components. Pulse coupled neural network is used to obtain useful information from the image.
MRI and CT	[33]	Brain	Hybrid image fusion	The image fusion is performed using principal component analysis and independent component analysis.
MRI and CT	[34]	Brain	Adolescent Identity Search Algorithm	The proposed approach decomposes the input image into high and low frequency component using nonsubsampled shearlet transform.
MRI and PET	[35]	Brain	Spectral Total Variation Transform	The proposed method decomposes the source image into base components and then combined using spatial frequency dual channel model.

**Table 2:** Performance evaluation of the proposed approach.

Fusion technique	Average structural similarity	Mutual information
Shift-invariant shearlet transform [37]	0.7104	2.2583
Wavelet transform [38]	0.6725	2.3171
Nonsubsampled shearlet transform [39]	0.8051	2.4336
Multilevel local extrema [40]	0.8175	2.5377
Proposed method	0.8551	2.8059

## Data Availability

The original contributions generated for this study are included in the article; further inquiries can be directed to the corresponding author.

## Abbreviations

MRI: Magnetic Resonance Image
PET: Positron Emission Tomography
GAN: Generative adversarial network
SPECT: Single-Photon Emission Computed Tomography
CT: Computed Tomography
HT: Hilbert Transform
IHS: Intensity Hue Saturation
CNN: Convolutional Neural Network
NN: Neural network.
